RETRACTED

# Evidence of Coal-Fly-Ash Toxic Chemical Geoengineering in the Troposphere: Consequences for Public Health

**DOI:** 10.3390/ijerph120809375

**Published:** 2015-08-11

**Authors:** J. Marvin Herndon

**Affiliations:** Transdyne Corporation, 11044 Red Rock Drive, San Diego, CA 92131, USA; E-Mail: mherndon@san.rr.com; Tel.: +1-858-271-4030; Fax: +1-858-271-1615

**Keywords:** geoengineering, coal fly ash, aerosol particulates, chemtrails, autism spectrum disorder (ASD), Alzheimer’s disease, Parkinson’s disease, attention deficit hyperactivity disorder (ADHD), neurological disorders, chemically mobile aluminum

## Abstract

The widespread, intentional and increasingly frequent chemical emplacement in the troposphere has gone unidentified and unremarked in the scientific literature for years. The author presents evidence that toxic coal combustion fly ash is the most likely aerosolized particulate sprayed by tanker-jets for geoengineering, weather-modification and climate-modification purposes and describes some of the multifold consequences on public health. Two methods are employed: (1) Comparison of 8 elements analyzed in rainwater, leached from aerosolized particulates, with corresponding elements leached into water from coal fly ash in published laboratory experiments, and (2) Comparison of 14 elements analyzed in dust collected outdoors on a high-efficiency particulate air (HEPA) filter with corresponding elements analyzed in un-leached coal fly ash material. The results show: (1) the assemblage of elements in rainwater and in the corresponding experimental leachate are essentially identical. At a 99% confidence interval, they have identical means (T-test) and identical variances (F-test); and (2) the assemblage of elements in the HEPA dust and in the corresponding average un-leached coal fly ash are likewise essentially identical. The consequences on public health are profound, including exposure to a variety of toxic heavy metals, radioactive elements, and neurologically-implicated chemically mobile aluminum released by body moisture *in situ* after inhalation or through transdermal induction.

## 1. Introduction

The interplay of political, military, and commercial interests during World War II led to the development and grand-scale deployment of a host of herbicides and pesticides such as dichlorodiphenyltrichloroethane (DDT). In her 1962 book *Silent Spring* [1] Rachel Carson called attention to the unintended consequences of herbicide and pesticide use, and launched the modern environmental movement. Half a century later there is growing evidence of a grave new and persistent global environmental health threat, again fomented by the interplay of political, military, and commercial interests. To date this new threat, posed by widespread, intentional tropospheric aerosol-particulate emplacement, has gone unremarked in the scientific literature for more than one decade. Here, based upon original research, the author discloses substantial evidence as to the identification and nature of the specific particulate substance involved and begins to describe the extent of this global public health and environmental threat.

RETRACTED

Recently there have been calls in both the popular and scientific press to begin discussions about the possibility of engaging in future stratospheric geoengineering experiments to counter global warming [2,3]. Geoengineering, also called weather-modification, has been carried out for decades at much lower altitudes in the troposphere. The recent calls for open discussion of climate control or geoengineering tend to obscure the fact that the world’s military and civilian sectors have modified atmospheric conditions for many decades as has been described by science historian, James R. Fleming [4]. Some of the early weather-modification research resulted in programs like Project Skywater (1961–1988), the U.S. Bureau of Reclamation’s effort to engineer “the rivers of the sky”; the U.S. Army’s Operation Ranch Hand (1961–1971), in which the herbicide Agent Orange was an infamous part; and its Project Popeye (1967–1971), used to “make mud, not war” over the Ho Chi Minh Trail. These few examples of weather-modification, all of them secret at the time they were engaged, show that the weather is in the words of the military, “a force multiplier” [5].

In the spring of 2014, the author began to notice tanker-jets quite often producing white trails across the cloudless blue sky over San Diego, California. The aerosol spraying that was happening with increasing frequency was a relatively new phenomenon there. The dry warm air above San Diego is not conducive to the formation of jet contrails, which are ice condensate. By November 2014 the tanker-jets were busy every day crisscrossing the sky spraying their aerial graffiti. In a matter of minutes, the aerosol trails exiting the tanker-jets would start to diffuse, eventually forming cirrus-like clouds that further diffuse to form a white haze that scattered sunlight, often occluding or dimming the sun. Aerosol spraying was occasionally so intense as to make the otherwise cloudless blue sky overcast, some areas of sky turning brownish (Figure 1). Sometimes the navigation lights of the tanker-jets were visible as they worked at night, their trails obscuring the stars overhead; by dawn the normally clear-blue morning sky already had a milky white haze. Regardless, aerosol spraying often continued throughout the day. The necessity for daily aerosol emplacement stems from the relatively low spraying-altitudes in the troposphere where mixing with air readily occurs bringing down the aerosolized particulates and exposing humanity and Earth’s biota to the fine-grained substance. The author’s concern about the daily exposure to ultra-fine airborne particulate matter of undisclosed composition and its concomitant effect on the health of his family and public health in general prompted the research reported here.

RETRACTED

**Figure 1:** Composite of four images of the blue sky over San Diego taken on cloudless days showing various instances of the on-going daily tanker-jet spraying of ultrafine-particulates into the troposphere. Upper Left: Spraying just started. Note that one tanker-jet turned off the spray in mid-flight. The “clouds” are dispersed particulates; Lower Right: Overcast “clouds” produced by intense tanker-jet emplacement of particulates.

Since the beginning of the 21st century there have been numerous observations of tanker-jet aerosol particulate spraying. Sometimes samples of rainwater, soil, and other residue were collected by concerned citizens and sent to commercial certified laboratories to be analyzed, although without an understanding of what tests should be made. The composition of the aerosolized particulate matter has been a tightly held secret. In the face of this unknown, there has been much sincere speculation in books and on the Internet, but also disinformation, attempts to convince the public that the particulate trails are nothing more than ice crystals formed from jet exhaust, and to pin on concerned citizens the pejorative moniker “conspiracy theorists”.

From the variety of observations reported in books and on the Internet, one might reasonably conclude that, at least during the early years, various weather-modification experiments were undertaken. But as indicated by photographic data and chemical analyses of post-spraying rainwater, one particular methodology was developed that ultimately was observed by the author to be operational on a daily basis in the skies over San Diego, and reportedly is now operational over much of the United States and in a number of foreign countries as well [6]. Beside the observational commonality, post-spraying rainwater was frequently found to contain aluminum and barium, two elements usually not present in naturally-occurring rainwater; sometimes strontium, a third element, was included in the tests and determined to be present [7]. The presence of strontium together with barium suggests that the undisclosed particulate matter is derived from a natural product, because alkaline earth elements, Group II on the Periodic Table, behave similarly and are often found together in nature. For example, cement contains calcium and often contains some strontium as well. That bit of insight evoked further considerations related to the potential costs and logistics of annually producing millions of tons of the undisclosed particulate matter and doing so out of public view.

RETRACTED

Industrial coal burning produces four types of coal combustion residuals (CCRs): fly ash, bottom ash, boiler slag, and flue gas desulfurization product (FGDP), *i.e.*, gypsum. Bottom ash is heavy and settles out; coal fly ash, on the other hand, is comprised of micron and sub-micron particles that would go up the smokestack unless captured and stored. Because of its well-known adverse environmental health effects, Western nations now mandate that coal combustion fly ash is to be captured and stored [8,9]. Representatives of coal burning utilities and their trade organizations actively promote commercial applications for coal fly ash, which, to name a few, include uses as additives to Portland cement, agricultural soil amendments, replacement for compacted backfills, mine reclamation, melting river ice, and as subsurface for roads. Some applications pose potential environmental health risks in the short term and/or in the long term as coal fly ash is a concentrated repository for many of the trace elements that were trapped in coal during its formation, including, but not limited to, arsenic, barium, beryllium, boron, cadmium, chromium, cobalt, lead, manganese, mercury, molybdenum, selenium, thallium, thorium, vanadium and uranium. 

Although seemingly unacknowledged in publicly accessible reports and in scientific literature as a potential material for geoengineering, coal fly ash is one major global waste product stream with the appropriate grain-size distribution for aerosolized tropospheric spraying that is readily available at extremely low cost and with existent processing and transport infrastructure. The author submits the following hypothesis: Coal fly ash is most likely the aerosolized particulate sprayed in the troposphere by tanker-jets for geoengineering, weather-modification and climate-modification purposes.

The objectives of the research are to provide substantial scientific evidence as to the correctness of the hypothesis, namely, that coal fly ash is the aerosolized particulate sprayed in the troposphere by tanker-jets for geoengineering, weather-modification and climate-modification purposes and to reveal some of the adverse human public health consequences and the antagonistic consequences on Earth’s environment and biota.

RETRACTED

## 2. Experimental Section

The methodology is two-fold: (1) Compare element ratios analyzed in rainwater, which were leached in the atmosphere from aerosolized particulates, with the corresponding element ratios that were extracted from coal fly ash into water in laboratory leaching experiments; and, (2) Compare the element ratios analyzed in dust collected outdoors on a HEPA filter with corresponding element ratios analyzed in coal fly ash material.

One of the reasons coal fly ash is sequestered, usually in lined ponds, is that a variety of toxic chemical elements are readily extracted by water, including but not limited to aluminum, arsenic, cadmium, chromium, thallium, lead, mercury and uranium. Scientists have conducted leaching experiments on coal fly ash samples, but none of the various investigations appear to be as thorough as that of Moreno *et al.* [10]. They obtained coal fly ash samples from 23 different European sources (from Spain, The Netherlands, Italy and Greece) which they analyzed for 33 chemical elements. They leached 100 grams of each coal fly ash sample with one liter of distilled water for twenty four hours, and then determined the concentrations of 38 elements in the leachate, the water-extract, from each experiment. Although there were some variations observed in the pre-leach coal fly ash chemical compositions and in the relative proportion of extracted elements in the leachate and variations in the resulting pH, the overall pattern of leachate elements was remarkably consistent among the different fly ash sources. Table 1 summarizes the average values for European coal fly ash pre-leach compositions and the average values of leachate chemical compositions that include those used in the present investigation.

**Table 1:** Average chemical composition of the 23 un-leached and leached (leachate) European coal fly ash samples from Moreno *et al.* [10].

Element	Un-Leached μg/kg	Leached (Leachate) µg/L	Element	Un-Leached µg/kg	Leached (Leachate) µg/L
Aluminum	7.00 × 10^4^	5.37 × 10^3^	Molybdenum	1.10 × 10^1^	3.66 × 10^−1^
Antimony	1.20 × 10^1^	3.60 × 10^−2^	Nickel	1.22 × 10^2^	1.68 × 10^−2^
Arsenic	7.06 × 10^1^	8.35 × 10^−2^	Niobium		6.22 × 10^−4^
Barium	1.38 × 10^3^	5.34 × 10^−1^	Phosphorus	1.22 × 10^3^	2.22× 10^2^
Beryllium	9.66	3.00 × 10^−4^	Potassium	1.43 × 10^4^	
Boron	2.38 × 10^2^	3.32	Rubidium	1.04 × 10^2^	3.04 × 10^−2^
Cadmium	1.87	7.61 × 10^−4^	Scandium		4.32 × 10^−3^
Calcium	4.03× 10^4^	3.48 × 10^5^	Selenium	2.24 × 10^1^	8.12 × 10^−2^
Cesium		2.78 × 10^−3^	Silicon	2.27 × 10^5^	6.57 × 10^3^
Chromium	1.54 × 10^2^	2.99 × 10^−1^	Sodium	2.98 × 10^3^	1.51 × 10^4^
Cobalt	4.13 × 10^1^	2.30 × 10^−3^	Strontium	1.09 × 10^3^	5.09
Copper	9.94 × 10^1^	6.97 × 10^−3^	Sulfur	3.78 × 10^3^	1.57 × 10^5^
Gallium		2.24 × 10^−2^	Thallium		4.61 × 10^−4^
Germanium	1.18 × 10^1^	6.20 × 10^−3^	Thorium	3.25 × 10^1^	9.83 × 10^−4^
Hafnium		1.01 × 10^−3^	Tin	8.48	6.96 × 10^−4^
Iron	2.89 × 10^4^	1.22 × 10^2^	Titanium	7.01 × 10^3^	4.27 × 10^−2^
Lead	1.29 × 10^2^	1.30 × 10^−3^	Uranium	1.34 × 10^1^	4.65 × 10^−4^
Lithium	1.95 × 10^2^	1.18	Vanadium	2.53 × 10^2^	1.18 × 10^−1^
Magnesium	1.02 × 10^4^	2.85 × 10^3^	Zinc	1.90 × 10^2^	2.70 × 10^−2^
Manganese	4.84 × 10^2^	4.35			

With its normally limited natural cloud cover San Diego is ideal for observing tanker-jet dispersal of ultra-fine particulates. Because the city lacks heavy industries and their particulate pollution, it is an ideal environment to ascertain by rainwater measurement the nature of the specific particulates being sprayed which are leached by rainwater. The author personally collected rainwater samples for chemical analysis and compared those data to corresponding average values of experimental leachate chemical analyses [10], which as shown below provides a firm basis for identifying the particulate substance being emplaced as an aerosol in the troposphere as coal fly ash. Because of persistent spraying, rainwater devoid of spray contamination was not available.

RETRACTED

For three months during a period of intense aerial spraying in 2011, an individual in Los Angeles, California captured and had analyzed outdoor air-borne particulates.The results were posted on the Internet [11]; subsequently the author obtained the analytical laboratory report. The requested analyses returned results for aluminum, barium and twelve trace elements. But the meaning of the data was not clear at the time. Comparison of those data with corresponding pre-leach average coal fly ash chemical analyses (Table 1), as shown below, further reinforces the correctness of identifying the particulate substance as coal fly ash that is being sprayed into the troposphere by tanker-jets for geoengineering.

## 3. Results and Discussion

The average elemental composition of each of the 38 elements from the 23 different sources of European coal fly ash leach studied by Moreno *et al.* [10], presented as ratios relative to aluminum, is shown in Figure 2 as a function of Atomic Number. Normalization to one common element, in this case aluminum, makes comparisons possible when total mass or total volume is not available. In this plot, the less abundant leachate element ratios are not shown. Note that aluminum (Atomic Number 13), strontium (38), and barium (56), elements which are sometimes determined in post-spraying rainwater, are relatively abundant.

**Figure 2:** The average leachate chemical concentration of each of the 38 elements from the 23 different sources of European coal fly ash (Table 1) studied by [10], normalized to aluminum so as to facilitate comparison with analyzed post-aerosol-spraying rainwater. Elements of lower concentration are not shown. Red leachate elements correspond to those measured in San Diego rainwater (Figure 3), from left to right, Boron, Magnesium, Aluminum, Sulfur, Calcium, Iron, Strontium and Barium.

RETRACTED

Two commercial state-of-California certified laboratories, Babcock Laboratories, Inc. and Basic Laboratory, were engaged for the San Diego rainwater analyses by inductively coupled plasma mass spectrometry. Their analytical results were consistent to within 2%–10%. Figure 3 shows concentrations of 8 chemical elements, normalized to aluminum, measured in post-aerosol-spraying San Diego rainwater for comparison with corresponding element ratios in the [10] water-extract of coal fly ash leaching experiments (Table 1).

**Figure 3:** The chemical concentrations of 8 elements, normalized to aluminum, measured in post-aerosol-spraying San Diego rainwater for comparison with similar average element ratios in the leachate of coal fly ash from Figure 1. This figure shows that post-spraying rainwater leached the same elements, in similar proportions, to the elements leached from coal fly ash in laboratory investigations [10]. This is strong evidence that the substance emplaced into the troposphere is coal fly ash. At a 99% confidence interval, the two sets of data have the same mean (T-test) and the same variance (F-test).

Like a fingerprint, the 8-element ratios of the San Diego rainwater extract of the tropospheric-emplaced particulate matter match element-by-element the laboratory water extract of coal fly ash within the range of observations. Said another way, the tropospheric-emplaced matter has the same water-leach characteristics as coal fly ash for at least eight elements, which is indeed strong evidence of the identification of the aerosolized substance as coal fly ash. For any indicated element the difference between the rainwater extract and average experimental coal fly ash element extract is less than the differences observed between the element extracted experimentally from the various coal fly ash sources [10]. 

Without mass or volume totals, statistical treatment was somewhat limited. Nevertheless, at a 99% confidence interval, the assemblage of elements in the rainwater and in the corresponding experimental leachate have identical means (T-test) and identical variances (F-test). Furthermore, the 8-element “fingerprint” shown in Figure 3 is comprised of elements with different chemical properties and thus provides extremely strong validation of the hypothesis: Coal fly ash is most likely the aerosolized particulate sprayed in the troposphere by tanker-jets for geoengineering, weather-modification and climate-modification purposes.

RETRACTED

One limitation in the use of commercial laboratories is in their limits of detection for some elements. Note from Figure 2 that the experimental coal fly ash leachate element ratios span six orders of magnitude. When academic research laboratories, with their high sensitivity capabilities, hopefully repeat the post-spray rainwater measurements, additional “matched pairs” for other elements will doubtlessly be added to the coal fly ash “fingerprint” presented in Figure 3.

For about fifteen years concerned individuals have sampled water, soil, and other materials in attempt to learn what is being sprayed into the atmosphere. From 15 May 2011 through 15 August 2011, a period intense tanker-jet spraying, an individual in Los Angeles, California operated a Honeywell model HHT081 HEPA Filter in her backyard in the vicinity of Olympic and La Cienega Boulevard, Los Angeles, California, 90035. Samples were collected and then transferred via chain-of-custody to American Scientific Laboratory, a state-of-California certified laboratory for analysis of aluminum, barium, and twelve trace elements by inductively coupled plasma mass spectrometry. 

Figure 4 shows concentrations of 14 chemical elements, normalized to aluminum, measured in the Los Angeles HEPA air filter dust for comparison with corresponding average element ratios for un-leached coal fly ash data (Table 1) from [10].

**Figure 4:** The chemical concentrations of 14 chemical elements, normalized to aluminum, measured in the Los Angeles HEPA air filter dust for comparison with corresponding average element ratios for un-leached coal fly ash (Table 1) data from [10]. This figure shows the 14 elements measured in the collected filter dust occur in the same relative proportions as similar elements in un-leached coal fly ash from published laboratory investigations [10]. This is strong evidence that the substance emplaced into the troposphere is coal fly ash. At a 99% confidence interval, the two sets of data have the same mean (T-test) and the same variance (F-test).

Like a fingerprint, the 14-element ratios of the HEPA dust match well the corresponding average chemical element ratios of un-leached coal fly ash. As with Figure 3 data, without mass or volume totals, statistical treatment was somewhat limited. Nevertheless, at a 99% confidence interval, the assemblage of elements in the HEPA dust and in the corresponding average coal fly ash have identical means (T-test) and identical variances (F-test). 

RETRACTED

Coal fly ash from difference sources vary somewhat in their relative proportions of chemical elements. Figure 5, a plot of the normalized high and low value for each of the 14 respective elements from un-leached coal fly ash [10], provides an indication of the range of variation in the coal fly ash material from different sources. Significantly, for any indicated element ratio in Figure 4, the difference between HEPA dust material and average coal fly ash composition is generally less than the extremes observed between high and low values of the various coal fly ash sources shown in Figure 5. Furthermore, the 14-element “fingerprint” shown in Figure 4 is comprised of elements with different chemical properties, implying a unique process, and thus further provides extremely strong validation of the hypothesis: Coal fly ash is most likely the aerosolized particulate sprayed in the troposphere by tanker-jets for geoengineering, weather-modification and climate-modification purposes.

**Figure 5:** This figure is a plot of the normalized high and low value for each of the 14 respective elements from un-leached coal fly ash [10]. It provides an indication of the range of variation in un-leached coal fly ash material from different sources. This natural variation in coal fly ash elemental compositions may help to explain the variations observed in Figure 3 and Figure 4.

Reliable observers have reported tropospheric aerosol emplacement since the late 1990s. In the early phases of the program one might suspect that a variety of substances were tried. At what point was coal fly ash chosen as the preferred substance? In the past, one of the great uncertainties about analyzing post-aerosol rainwater has been which elements to measure. Aluminum was commonly measured, while barium and strontium were sometimes measured; other chemical elements were rarely measured. As aluminum, barium and strontium are prominent water-extracts of coal fly ash, their presence in post-aerosol rainwater might be taken as a 3-element fingerprint of aerosolized coal fly ash, albeit with much less certainty than the 8-element fingerprint shown in Figure 3. Based upon the 3-element fingerprint, with its limited certainty, the year 2002 is the earliest data found to date showing simultaneous measurement of these three elements in post-aerosol rainwater [12]. Within that certainty-limitation, the 3-element fingerprint in post-spraying rainwater measurements indicates the global extent of tropospheric aerosol coal fly ash dispersing: such measurements have been made in the United States, Canada, France, Portugal, Germany, Australia, and New Zealand. Further, this list is unlikely to be exhaustive. The global extent of tropospheric coal fly ash emplacement is inferred from rainwater analyses reporting the three elements (aluminum, barium and strontium) that are prominent in the leachate of laboratory coal fly ash water-leach experiments.

RETRACTED

The research reported here provides strong evidence that coal fly ash is the aerosolized particulate sprayed in the troposphere by tanker-jets for geoengineering, weather-modification and climate-modification purposes. The evidence presented warrants discussion as to (1) what additional investigations should be undertaken to confirm further the identity of coal fly ash as the aerosolized particulates, (2) the consequences of troposphere-emplaced coal fly ash on public health and on Earth’s biota, and (3) the resultant geophysical implications.

The rainwater and dust sample collection, in San Diego and Los Angeles, respectively, took place in areas far removed from aerosol-polluting heavy industries under circumstances of intense and persistent aerial spraying of fine grain particulates that left a white haze in the sky. The tropospheric lifetime of the particulates was sufficiently short as to necessitate near-daily spraying, which is an argument against the collected samples originating far away, such as from China due to the global movement of weather. Whereas the “fingerprint” evidence is compelling, strongly suggesting identical processes/materials, additional investigations should be undertaken and, indeed, are being planned.

Off the coast of Southern California individuals have observed tanker jets “dumping” massive quantities of particulate matter in relatively short bursts, colloquially called “bombs”, which disperse significantly before prevailing winds bring the matter to the coast line. One plan under consideration is to use aircraft to capture in flight some of the concentrated material, which would then be analyzed physically and chemically, and as well be subjected to leaching experiments. 

In the 1970s acid rain [13] liberated aluminum in a chemically mobile form from otherwise inert sources, such as mine tailings, that posed an environmental health threat to a host of organisms [14,15]. Forest die-offs, reduced survival or impaired reproduction of aquatic invertebrates, fish, and amphibians were directly connected to aluminum toxicity, while indirect effects on birds and mammals were also identified [16]. Tropospheric aerosolized coal fly ash poses a similar environmental health threat without necessarily requiring an acid environment. In the experiments by Moreno *et al.* [10], distilled water led to aluminum extraction while other chemical reactions yielded leachate pH values in the range 6.2–12.5. The pH of post-spraying rainwater is a function of the composition of the coal fly ash and the degree of its equilibration with atmospheric water. Natural rainwater has an acidic pH of about 5.7 due to interaction with atmospheric CO_2_ [17]. The pH of the analyzed post-spraying San Diego rainwater was 5.2 whereas in instances elsewhere it has been observed as high as 6.8.

RETRACTED

Long exposure to air pollution particulates, not necessarily coal fly ash, in sizes ≤ 2.5µm (PM_2.5_) is associated with morbidity and premature mortality [18,19]. One may therefore reasonably conclude that aerosolized coal fly ash, at least the PM_2.5_ component, is detrimental to human health.

The ultra-fine particles of aerosolized coal fly ash do not remain at tanker-jet operational altitudes: they mix with and pollute the air people breathe. Tropospheric aerosol coal fly ash can potentially endanger humans through two primary routes: (1) ingestion of rainwater-extract of coal fly ash toxins, directly or after concentration by evaporation and (2) particulate intake through inhalation or through contact with the eyes or skin [20]. In the latter instance, harm to humans can arise from *in situ* body-fluid extraction of coal fly ash toxins [21] as well as from the consequences of tissue contact [22]. Coal fly ash that is PM_2.5_ is readily entrained in terminal airways and alveoli and retained in the lungs for long periods of time; the small grain size enables it to penetrate and reach deep within the airways where it can cause inflammation and pulmonary injury [23].

Coal fly ash contains a host of potentially leachable toxins, including aluminum, arsenic, barium, beryllium, boron, cadmium, chromium (III), chromium (IV), cobalt, lead, manganese, mercury, selenium, strontium, thallium, thorium, and uranium. Coal fly ash has been described as being more radioactive than nuclear waste [24]. Moreover, many of the most toxic elements are enriched in the PM_2.5_ component of coal fly ash [25]. Whether or not the coal fly ash used for geoengineering is selectively enriched in PM_2.5_ is not known, but enrichment in the small particle size fraction would be advantageous in yielding greater surface area for sunlight reflection.

The extent of adverse health consequences from aerosolized coal fly ash depends on a variety of factors including age, physical condition, individual susceptibility, concentration and exposure duration. Moreover, some toxic elements from tropospheric spraying of coal fly ash, in addition to direct bodily input by inhalation or transdermal infusion, may be concentrated by processes in nature. Arsenic, for example, one of the coal fly ash toxins, poses the greatest health threat in its inorganic form. Arsenic can be taken up by a variety of organisms and, like mercury, can be passed up the food chain [26]. Arsenic can be involved with hypertension-related cardiovascular disease [27], cancer [28], stroke [29], chronic lower respiratory diseases [30] and diabetes [31]. Arsenic leached from coal fly ash taken in by pregnant women can crossover the placenta to the fetus [32]. Concentration and exposure duration increase likelihood of this happening. 

RETRACTED

The evidence presented here of deliberate, widespread and pervasive spraying of coal fly ash into the troposphere, which mixes with the air people breathe, opens new research possibilities into the physiological effects of long-term exposure to a substance that potentially releases multifarious toxins upon exposure to internal body fluids. Those subjects are beyond the scope of the present article. Nevertheless, mention should be made of perhaps the least appreciated coal fly ash potentially water-extracted toxin, chemically mobile aluminum.

Although aluminum is abundant in the Earth’s crust, it is highly immobile. Consequently, our planet’s biota, including humans, have not developed natural defense mechanisms for exposure to chemically mobile aluminum. It is a matter of grave concern that aluminum in a chemically mobile form can be readily extracted from coal fly ash with rainwater or *in situ* with body fluids. Aluminum is implicated in such neurological diseases as autism spectrum disorder (ASD), Alzheimer’s disease, Parkinson’s disease, and attention deficit hyperactivity disorder (ADHD) [33,34,35,36,37] all of which have markedly increased in recent years. Aluminum is thought to impair fertility in men [38] and is also implicated in neurological disorders of bees and other creatures [39,40,41].

If in fact some instances of neurological diseases are related to weather-modification activities during the last two decades involving the tropospheric coal fly ash aerosols, then the recent ramp-up in tanker-jet spraying, as witnessed by this author in San Diego, will likely cause a sharp spike in their occurrence. Epidemiological investigations of wide-ranging scope, including for example childhood and elderly disorders and birth defects, may begin to shed light on the human toll extracted by spraying coal fly ash into the troposphere. Those investigations should especially consider airline flight crews and frequent airline travelers who breathe the air at nearly the same altitude as the spraying.

The near-daily intense aerial spraying over San Diego witnessed by the author is part of a multinational Western, if not global, program that has been observed for a number of years in United States, Canada, Europe, Australia and New Zealand, but never acknowledged publically by officials. Without public candor it is difficult to know the underlying motivations and the range of specific activities involved. One thing seems certain: the potential damage to public health and the environment is likely to be unprecedented in its planetary scope. 

RETRACTED

The process of burning coal concentrates the impurities in coal fly ash, an unnatural anhydrous chemical complex whose environmental health hazards are well-known. For decades individuals and organizations have fought long and hard for regulations requiring sequestration of this hazardous industrial waste product. So what, one might ask, is the reason for the current, widespread, pervasive spraying of coal fly ash into the troposphere with its potential harm to public health and the environment? 

Since the United Nations Intergovernmental Panel on Climate Change (IPCC) was established in 1988 there has been much interest in global warming, which is perceived as a security threat. Geoengineering offers two basic approaches to the problem of global warming: Remove and trap carbon dioxide, or block sunlight from reaching the Earth. Trapping carbon dioxide is a difficult, prohibitively expensive, undeveloped technology. Blocking sunlight is almost universally recognized by geoengineers as being relatively inexpensive, easy to implement, and moreover has a precedent in nature: major volcanic eruptions inject ash into the upper atmosphere (stratosphere) which may remain suspended for a year or more, dimming sunlight and momentarily cooling Earth. 

While academicians debate geoengineering as an activity that might potentially be needed in the future [2,3], evidence suggests that Western governments/militaries moved ahead with a full scale operational geoengineering program. But instead of mining and milling rock to produce artificial volcanic ash in sufficient volumes to cool the planet, they adopted a low-cost, pragmatic alternative, but one with consequences far more dire to life on Earth than global warming might ever be, and used coal combustion fly ash. To make matters worse, instead of placing the material high into the stratosphere, where there is minimal mixing and the substance might remain suspended for a year or more, they opted to spray coal fly ash into the lower atmosphere, the troposphere, which mixes with the air people breathe and gets rained down to ground.

Aside from the serious potential toxicity ramifications on public health and Earth’s biota that derive directly from aerosolized emplacement of coal fly ash into the troposphere, such pervasive, widespread, tanker-jet spraying affects weather and Earth’s heat balance in ways that act in opposition to cooling the Earth. Those who reside in locations where natural cloud cover is rare, like San Diego, notice the rapid cooling after the sun goes down, except on cloudy days when heat is retained. During the daytime coal fly ash clouds may block sunlight, but at night may retard heat loss from the Earth, act to prevent rainfall, and contribute to global warming. Nighttime tanker-jet spraying, presumably to the hide the activity from public view, further retards heat loss.

RETRACTED

There is yet another consequence of tropospheric coal ash spraying that is contrary to cooling the Earth and has potentially far-reaching adverse ecological and public health implications: weather modification and concomitant disruption of habitats and food sources. As reported by NASA, “Normal rainfall droplet creation involves water vapor condensing on particles in clouds. The droplets eventually coalesce together to form drops large enough to fall to Earth. However, as more and more pollution particles (aerosols) enter a rain cloud, the same amount of water becomes spread out. These smaller water droplets float with the air and are prevented from coalescing and growing large enough for a raindrop. Thus, the cloud yields less rainfall over the course of its lifetime compared to a clean (non-polluted) cloud of the same size” [42]. In addition to preventing water droplets from coalescing and growing large enough to fall to Earth, coal fly ash, which formed under anhydrous conditions, will hydrate, trapping additional moisture thus further acting to prevent rainfall. That may cause drought in some areas, floods in others, crop failure, forest die-offs, and adverse ecological impacts, especially in conjunction with the chemically-mobile-aluminum contamination from coal fly ash. The consequences ultimately may have devastating effects on habitats and reduce human food production.

## 4. Conclusions

The original research reported here provides strong evidence for the correctness of the hypothesis: Coal fly ash is most likely the aerosolized particulate sprayed in the troposphere by tanker-jets for geoengineering, weather-modification and climate-modification purposes. That evidence is based upon the discovery that: (1) the assemblage of 8 elements in rainwater and in the corresponding experimental leachate are essentially identical. At a 99% confidence interval, they have identical means (T-test) and identical variances (F-test); and, (2) the assemblage of 14 elements in the HEPA dust and in the corresponding average un-leached coal fly ash are likewise essentially identical.

RETRACTED

Evidence indicates that tropospheric spraying of coal fly ash (1) has been taking place throughout the 21st century, (2) on an international scale, and (3) with significant ramping-up since about 2013. Throughout that period of time there has been a program of well-orchestrated disinformation, but no public disclosure, no informed consent, and no public health warnings.

The profound implications on environmental health include exposing humans and Earth’s other biota to: (1) chemically mobile aluminum, implicated in neurological disorders and botanic demise; (2) exposure to toxic heavy metals and radioactive elements; (3) preventing rainfall with concomitant loss of food production and habitats; and, (4) possibly contributing to global warming with concomitant arctic melting.

More than a half century ago Rachel Carson called the world’s attention to the unintended consequences of herbicides and pesticides widely employed by agriculture. Instead of turning a blind eye, people everywhere became motivated to stop the worst of this environmental onslaught. Today we are fully aware of the vast interconnected web of dependencies and symbioses that comprise life on our planet. Earth exists in a state of dynamic biological, chemical, and physical equilibrium whose complexity far exceeds the understanding of contemporary science. The pervasive tropospheric spraying of coal fly ash threatens this equilibrium, whose delicacy or whose resilience we cannot quantify. Human health is at risk as is Earth’s biota. Are we to remain silent? Or will we exercise our primal right to speak in our own defense as a species and question the sanity of emplacing coal fly ash in Earth’s perpetually moving atmosphere?
